The article "Investigations on the Changes of Serum Proteins in Rabbits after Trimeresurus stejnegeri Venom Injection via Mass Spectrometry-Based Proteomics" was retracted in 2023. Reasons: signs of a paper mill; suspected computer-generated content; unreliable results or conclusions; concerns about the data.

# Investigations on the Changes of Serum Proteins in Rabbits after *Trimeresurus stejnegeri* Venom Injection via Mass Spectrometry-Based Proteomics

**DOI:** 10.1155/2022/9239662

**Published:** 2022-06-24

**Authors:** Shijun Wang, Weilian Yang, Wanling Shi, Fuwei Chen, Fanghua Shen, Meiji Zhang, Qiuxiang Su, Chao Shi, Qinyao Yu, Tao Chen

**Affiliations:** Surgery of Traditional Chinese Medicine, People's Hospital Affiliated to Fujian University of Traditional Chinese Medicine, Fuzhou 350004, Fujian, China

## Abstract

**Purpose:**

There are few studies on protein phosphorylation in the process of snake poisoning. The purpose of this study was to investigate the toxic mechanism of *Trimeresurus stejnegeri* at the protein level by determining the differential expression of phosphorylated proteins in rabbits after poisoning using proteomics.

**Methods:**

The *Trimeresurus stejnegeri* venom model in rabbits was established by intramuscular injection of 20 mg/kg venom. The serum was collected and the differential expression of phosphorylated proteins in the serum was determined by the iTRAQ technology, TiO2 enriched phosphorylated peptides, and the mass spectrometry analysis. The functional analysis was conducted using ClueGO software and the related mechanism was evaluated by the network analysis of biological interaction. The expression level of related proteins was determined by the Western blotting assay.

**Results:**

Compared to the control group, 77 differentially expressed proteins were observed in the model group. These proteins were closely associated with the complement and agglomerate cascade signaling pathways, the HIF signaling pathway, the pentose phosphate pathway, and the cholesterol metabolism signaling pathway. According to the results of network analysis, TF and SCL16A1 were determined as the core proteins, which were identified by the Western blotting assay.

**Conclusion:**

The present study provided valuable phosphorylation signal transduction resources for investigating the toxic mechanism and the therapies for *Trimeresurus stejnegeri* poisoning.

## 1. Introduction

Snake poisoning is a serious public health issue in the tropical and subtropical countries of Africa, Asia, and Latin America [1]. The clinical responses of snake poisoning include respiratory arrest, obstruction of hemostasis, bleeding, and tissue damage [2]. Approximately, 80 thousand people die of snake poisoning and 0.3 million people suffer from amputation or permanent disability due to snake poisoning [3]. In response to the severity of snake poisoning [4], the World Health Organization (WHO) has made a plan to decrease the mortality and disability induced by snake poisoning by 50% before the year 2030, which includes the awards for the investigations on the next generation of therapy [5], which need the support of molecular mechanism of toxicity physiopathology using optimized representational methods. However, currently, the investigations on the protein phosphorylation during snake poisoning are rare.

The phosphorylation of proteins is one of the most basic, common, and important mechanisms for the regulation of protein activities and functions [6, 7]. The initiation or close of multiple types of biochemical functions can be regulated by the phosphorylation of proteins, such as the transcription and translation regulation, signal transduction, DNA damage repair, cell metabolism, secretion, and homeostasis [8]. The abnormal phosphorylation of proteins is closely associated with the development of several diseases and the production of protein phosphorylation is regarded as the sign of an abnormal state in an organism [9]. Therefore, the study of phosphorylated proteins in blood samples after snake venom poisoning is helpful to elucidate the related pathophysiologic mechanisms. It is widely reported that protein phosphorylation plays an important regulatory role in the process of poisoning [10]. Some protein kinases impact the structure and function of important organs by regulating complement activation, inflammatory responses, and immune interactions, which are also involved in the pathological poisoning processes [11]. Currently, the proteomic investigations on the serum and venom have been partly reported [12]. However, the research studies on the protein phosphorylation induced by snake venom poisoning are rare.

The present study identified the differentially expressed phosphorylated proteins post-snake venom poisoning through the high throughput method and conducted the proteomic investigation by the iTRAQ technology, method of TiO2 enriched phosphorylated peptides, and the mass spectrometry analysis. The present study revealed the important role phosphorylated proteins play in the toxic mechanism underlying snake venom poisoning and provided the basis for the future research studies on the pathological mechanism and the treatment strategies against snake venom poisoning.

## 2. Materials and Methods

### 2.1. The Establishment of the *Trimeresurus stejnegeri* Poisoning Rabbit Model

The Japanese rabbits were purchased from the Charles River Laboratories (Beijing, China) and the *Trimeresurus stejnegeri* venom was purchased from Fuzhou Wanlong Biotechnology Co., LTD (Fujian, China). After adapting for 7 days, rabbits were intramuscularly injected with 1.5 mg/kg, 2 mg/kg, 2.5 mg/kg, 11.5 mg/kg, 20 mg/kg, and 40 mg/kg *Trimeresurus stejnegeri* venom, respectively. The initial toxic dose was found to be 20 mg/kg, which was used as the dosage to establish the *Trimeresurus stejnegeri* poisoning rabbit model. Animals in the model group (*n* = 6) were injected with 20 mg/kg *Trimeresurus stejnegeri* venom and those in the control group (*n* = 6) were injected with the equal volume of normal saline. The blood was collected from the heart 4 hours later and the serum was separated, which was used for proteomics analysis and Western blot identification. This study was approved by the Ethics Committee of People's Hospital Affiliated to Fujian University of Traditional Chinese Medicine (FTCM2022-011).

### 2.2. The Isolation and Quantification of Proteins

40 *μ*L serum for each sample was collected and diluted with 360 *μ*L binding buffer. After loading the binding buffer, the column was placed in the collecting tube, followed by loading the samples. Then, the column was washed with 600 *μ*L binding buffer twice, followed by collecting the elution fractions and vacuum freeze-drying. The dried sample was resuspended with 300 *μ*L SDS buffer, followed by centrifugation at 12000 g for 10 min at the room temperature. The supernatant was collected and the proteins were quantified using the commercial BCA kit (CW0014S, CWBIO, Jiangsu, China).

### 2.3. SDS-PAGE Separation

For each sample, 10 *μ*g protein was collected and separated by 12% SDS-PAGE, followed by Coomassie blue staining using the eStain LG (L00755 C, Genscript, Jiangsu, China). The stained gel was imaged using the automatic digital gel image analysis system.

### 2.4. Enzymatic Hydrolysis of Trypsin

For each sample, 200 *μ*g protein was collected and added with 5 mM DTT solution, followed by incubation for 30 min under 55°C. The sample was cooled down on ice to room temperature. Then, the sample was added with 10 mM iodoacetamide and placed in the dark for 15 min at room temperature, followed by adding 6-fold volume acetone to precipitate the proteins. After being placed under −20°C for 4 hours, the sample was centrifugated at 8000 g for 10 min under 4°C to collect the precipitate, followed by volatilizing the acetone for 2-3 min. Approximately, 100 *μ*L TEAB (200 mM) was used to resuspend the precipitation and 1 mg/mL Trypsin-TPCK was added for digestion at 37°C overnight, followed by freeze-drying and storage at −80°C.

### 2.5. Peptide Tagging

Freeze-dried samples were added with 200 *μ*L 100 mM TEAB buffer in 1.5 mL EP tubes. TMT marker reagents (90061, Thermo Fisher) were added with 41 *μ*L anhydrous acetonitrile and then were added into samples and placed at room temperature for 1 hour. Subsequently, 16 *μ*L 5% hydroxylamine was added and incubated for 15 min to terminate the reaction, followed by freeze-drying and storage at −80°C.

### 2.6. The Enrichment of Phosphorylated Peptides

The freeze-dried peptides were suspended in 200 *μ*L Binding/Wash Buffer and the chromatographic column was placed into a 2 mL microcentrifuge tube, followed by centrifugation at 1000 g for 30 s to remove the storage buffer. The chromatographic column was placed in the binding phosphorylated peptides, followed by adding 200 *μ*L suspended peptide sample into the balanced centrifugal column. After incubation for 30 min, the chromatographic column was placed into the microcentrifuge tube, followed by centrifugation at 1000 g for 30 s. The column was washed using 200 *μ*L Binding/Wash Buffer three times and the phosphorylated peptides were enriched in the chromatographic column.

### 2.7. Chromatographic Conditions

The samples were loaded into the Acclaim PepMap100 (100 *μ*m × 2 cm, RP-C18, Thermo Fisher) at a speed of 300 nL/min, followed by being separated by Acclaim PepMap RSLC (75 *μ*m × 15 cm, RP-C18, Thermo Fisher). The mobile phase A was H_2_O-FA (99.9 : 0.1, v/v) and the mobike phase B was ACN-H_2_O-FA (80 : 19.9 : 0.1, v/v/v). The gradient elution condition was as follows: 0∼82 min, 5%–44% B; 82∼84 min, 44%–90% B; 84∼90 min, 90% B.

### 2.8. Mass Spectrometry Conditions

Under the positive ion mode, the mass resolution of the primary mass spectrometry was settled as 60000 and the automatic gain control value was settled as 1e6. The mass spectrometry scanning was settled as full scan with the range of m/*z* from 300 to 1600, which was used to scan the top 20 peaks. All MS/MS spectra were collected using a data-dependent high-energy collision cleavage under the positive ion mode. The collision energy was set as 32 and the resolution ratio of MS/MS was set as 30000. The automatic gain control value was settled as 2e5 and the dynamic exclusion time was set as 30 s.

### 2.9. The Analysis and Evaluation on the MS Database

ProteinPilot Software v.4.5 (AB Sciex, Framingham) was used to conduct the protein identification and quantification analysis on the MS/MS data. MaxQuant was used to search and identify peptides and analyze the relative quantitation.

### 2.10. Western Blot Analysis

Total proteins were isolated from HBMECs using the lysis buffer and quantified with a BCA kit (Takara, Tokyo, Japan). Proteins were loaded and separated by the 12% SDS-PAGE and were transferred to the PVDF membrane (Takara, Tokyo, Japan). After being incubated with 5% skim milk, the membrane was incubated with the primary antibody against SLC16A1 (1 : 1000, bs-10249R, Bioss, Beijing, China), p-SLC16A1 (1 : 100, AF7044, Affinity, Melbourne, Australia), TF (1 : 1000, bs-4690R, Bioss, Beijing, China), p-TF (1 : 100, AF7223, Affinity, Melbourne, Australia), and GAPDH (1 : 800, Abcam, Cambridge, UK), followed by being incubated with the secondary antibody (1 : 800, Abcam, Cambridge, UK) at room temperature for 1.5 hours. Finally, the ECL solution was used to visualize the bands, which were quantified by the Image J software.

### 2.11. The Motif Analysis on the Phosphorylation Site

Amino acid sequence motifs were analyzed by online software MoMo (https://meme-suite.org/meme/tools/momo) and the *p* value threshold was set as 10^−6^ (Modification Motifs, version 5.1.1).

### 2.12. Bioinformatics Analysis

Gene Ontology (GO) annotation analysis was performed using the UniProt-GOA database (https://www.ebi.ac.uk/GOA/). First, we convert the identifiable protein ID to UniProt ID, then match with the GO ID, and then obtain the relevant information according to the GO ID. If the UniProt-GOA database is not included, we use the ClueGO software to analyze the protein GO function. GO annotation analysis was performed from three aspects: biological process, cellular components, and molecular functions. Protein pathways are annotated using the KEGG pathway database: KEGG's online service tool KAAS is used to annotate the submitted proteins, and then, the annotated proteins are matched to the corresponding pathways through the KEGG mapper.

### 2.13. Construction of the Protein-Protein Interaction (PPI) Network

Through the interactive gene retrieval tool STRING (https://cn.string-db.org), a protein-protein interaction (PPI) network was constructed for genes with a significant differential expression. Discrete points in the network and other parameters are default. The PPI network is visualized in Cytoscape3.8.2 software (https://cytoscape.org). The cytoHubba network analysis plugin is used to calculate the degree of connection between proteins, and the greater the degree value is, indicating more interacting protein nodes, the greater the impact on the network, and the core genes of the PPI network were screened out.

### 2.14. Statistical Analysis

Data were expressed as mean ± SD and the data analysis was conducted using the GraphPad software. The Student's *t*-test was used to analyze data between 2 groups and the one-way ANOVA method was used for the analysis among groups. *p* < 0.05 was considered a significant difference.

## 3. Results

### 3.1. The Determination of the Optimized Poison Dosage

After injecting different dosages (1.5 mg/kg, 2 mg/kg, 2.5 mg/kg, 11.5 mg/kg, 20 mg/kg, and 40 mg/kg) of the *Trimeresurus stejnegeri* venom, no significant injury or death was observed in low-dose groups (1.5 mg/kg, 2 mg/kg, and 2.5 mg/kg). However, in high-dose groups (11.5 mg/kg, 20 mg/kg, and 40 mg/kg), the activity of rabbits was inhibited and swollen posterior limbs and paralysis were observed 30 min post-dosage. One-hour post-dosage, the rabbit's lips turned purple and eyes turned black. Animals in the 40 mg/kg group were found convulsive and dead 4 hours post-dosage. Rabbits in the 20 mg/kg group were dead 5 hours post-dosage and animals in the 11.5 mg/kg group were found dead 24 hours post dosing. Therefore, 20 mg/kg was chosen as the injection dosage. In poisoned rabbits, a bruise was observed at the injection site and relatively pale lung tissues were observed. No obvious pathological changes were observed in other organs.

### 3.2. The Quantification of Proteins in the Model and Control Groups

As shown in Table 1, there was no significant difference on the protein concentration between the model group and the control group.

### 3.3. Correlation Analysis for Protein Identification

The principal component analysis (PCA) was conducted to present the correlation between control and model in different dimensions. As shown in Figure 1, each dot represented the result of one repeat and the color represented different groups. A significant difference was observed between the control and the model groups as 2 sets of coordinate points were located relatively far away on the score chart, which obviously separated into 2 clusters.

### 3.4. Statistical Results of Differentially Expressed Proteins

Data with at least two nonnull values in three repeated experimental data were screened for statistical analysis. The standard for significant differentially expressed proteins was defined as follows: the expressional difference multiple was higher than 1.5 and the *p* value was lower than 0.05. The number of differentially expressed proteins between the control and model group was 77, among which 34 proteins were significantly upregulated and 44 proteins were significantly downregulated (as shown in supplementary materials).

### 3.5. The Screening Results of Differentially Expressed Proteins

The volcano plots were drawn using the multiples of protein expressional differences and the *p* value calculated from *t* test between the control and model groups. As shown in Figure 2, in the abscissa, the farther the distance to 0 point, the higher multiples of protein expressional differences were observed on the protein expression. On the ordinate, the farther the distance from 0 point, the more significant difference was observed in the protein expression. The red dots represent upregulation and blue dots represent downregulation. The gray dots represent proteins with no significant expression difference.

### 3.6. The Motif Analysis on the Phosphorylation Site

Motif is the pattern that protein kinases specially recognize residues, which represents the substrate bias of kinases. MOMO software was used to analyze the motif of the differential phosphorylation sites. In the tested 462 phosphorylated peptides, 567 phosphorylated sites located in 224 proteomes were found to be differentially expressed between 2 groups.

### 3.7. The Results of GO Analysis

According to the results of software analysis, the functions of 77 differentially expressed proteins were mainly involved in the following biological progressions: immune response, regulation of blood coagulation process, intracellular ion homeostasis, regulation of complement activation, and positive regulation of cellular transcriptional translation. Most differentially expressed proteins were found to be involved in extracellular regulatory processes and the next most differentially expressed proteins were found to be involved in the regulation of serine endopeptidase activity and calcium ion regulation processes. The results of GO analysis are shown in Figure 3.

### 3.8. The Results of KEGG Pathway Enrichment Analysis

As shown in Figure 4, entries with larger bubbles contained more differentially expressed proteins. The *p* value became smaller as the color of the bubble changed from red-green-blue-purple, which indicated more significant differences. Differentially expressed proteins were mainly involved in the following pathways: the regulation of complement system, HIF-1 signaling pathway, glycolysis and glycogenesis, iron death, and cholesterol metabolism pathways. Most differentially expressed proteins were found to be involved in the regulation of the complement system and the HIF-1 signaling pathway, which might be key related pathways responsible for the snake venom injury.

### 3.9. The Results of Protein-Protein Interaction (PPI) Analysis

According to the prediction of STRING database and the analysis of Cytoscape software, the circle represented the differentially expressed proteins and the size of the circles represented the degree of connectivity between 2 proteins. As shown in Figure 5, PPIs involved in differentially expressed proteins mainly focused on hemolysis proteins, immune regulatory proteins, and extracellular matrix regulatory proteins.

### 3.10. The Verification Results of TF and SLC16A1

As shown in Figure 6, the expression level of TF and SLC16A1 selected from differentially expressed proteins was further verified by western blot. Compared to the control group, p-TF/TF was significantly upregulated in the model group. In addition, compared to the control group, the expression level of p-SLC16A1/SLC16A1 was found significantly suppressed in the model group (*p* < 0.05). As an important coagulation factor, TF plays a catalytic role in cell coagulation by regulating microparticles (MPs). While SLC16A1 is a functional membrane protein, the downregulation of SLC16A1 is reported to induce the decline of cognitive function. Therefore, we speculate that TF and SLC16A1 may serve as candidate biomarkers for snake venom poisoning injury and prognosis.

## 4. Discussion

Currently, investigations on phosphorylated proteomics in the serum post-infection with the *Trimeresurus stejnegeri* venom are rare. To explore the pathological mechanism underlying the poisonousness induced by the *Trimeresurus stejnegeri* venom, the expression changes of protein phosphorylated protein spectrum in the peripheral circulatory system were compared between the model group and the control group. In the tested 462 phosphorylated peptides, 567 phosphorylated sites located in 224 proteomes were found to be differentially expressed between 2 groups. This study found that the number of differentially expressed proteins between the control group and the model group was 77 after induced by the *Trimeresurus stejnegeri* venom, which mainly involved the following biological processes: immune response, regulation of blood coagulation process, intracellular ion homeostasis, regulation of complement activation, and positive regulation of cellular transcriptional translation. Identified key factors, tissue factor (TF), and solute carrier family 16 member 1 (SLC16A1) were verified as potential biomarkers of snake venom poisoning, which were beneficial for monitoring the therapeutic efficacy against snake venom poisoning.

Utilizing different analysis software, several regulatory pathways were identified, such as the regulation of complement system, HIF-1 signaling pathway, glycolysis and glycogenesis, iron death, and cholesterol metabolism pathway. It is reported that the clinical characteristic of overactivation of certain complement-mediated inflammatory conditions is observed during the poisonous process of a snake bite [13]. Research studies indicate that snake venom components interact with complement proteins [14], and snake venom has been proved to initiate or aggravate the activation of proteins [15]. In addition, venoms originated from different snakes, such as *Trimeresurus stejnegeri*, spearhead vipers, and coral snakes, have been evidenced to trigger complement activation in normal human serum, which contributes to the production of anaphylatoxin and the assembly of soluble terminal complement complexes [16]. In the present study, we also found that in the results of differential protein enrichment analysis, the regulation on the complement system was the main function involved. In addition, snake venom poisoning also often results in severe hemorrhagic effects. However, the underlying mechanism is rarely reported. Our analysis indicated that in total differentially expressed proteins, the expressional changes of coagulation associated proteins were significant. As an important coagulation factor, TF functions as the catalyzer for cellular coagulation by regulating the microparticles (MPs) [17]. Our results showed that in the model group, p-TF was found significantly upregulated, which might be one of the key targets responsible for bleeding in rabbits post-snake venom poisoning.

What we were interested in were key pathways involved in the metabolic processing post-snake venom poisoning. In our previous research results, it was found that the expression level of SLC16A1 protein was significantly increased in the rabbit model exposed to snake venom, which was inconsistent with our experimental results. This may be due to individual differences. In previous experiments, we did not mix rabbit serum for mass spectrometry. SLC16A1 is a functional membrane protein and the downregulation of SLC16A1 is reported to induce the decline of cognitive functions [18]. In addition, it is reported that SLC16A1 is enriched in the neuron- and synapse-related pathways, indicating that SLC16A1 might be involved in the signal transduction of stress reaction and neuroprotection [19]. Apart from the neuroprotection function, SLC16A1 is reported to be closely associated with the energy metabolism-related progressions, such as lactic acid transport, pyruvate metabolism, and the citric acid cycle [20]. SLC16A1 is one of the genes that were significantly enriched in response to extracellular stimuli as SLC16A1 regulates the oxidative metabolism mediated by gluconeogenesis and lipogenesis [21]. Our results showed that p-SLC16A1 and SLC16A1 were both downregulated in the model group, indicating that the significant metabolic disorders in proteins, cholesterol, fatty acids, and glucose in rabbits were induced by large dosages of snake venom, which not only induced the injury on neurons and cognitive function but also impacted the normal metabolic progression. The disorders in coagulation and metabolism indicated that severe damages on the coagulation function and transport ability of the host were induced by the *Trimeresurus stejnegeri* venom and the key central network proteins were TF and SLC16A1. Therefore, TF and SLC16A1 could be used as the biomarkers candidates for the injury and prognosis of snake venom poisoning.

Taken together, valuable clues could be provided for the treatment and prognosis alleviation after snake venom poisoning by investigating the changes in phosphorylated proteomics in the rabbit peripheral circulatory system after injecting the *Trimeresurus stejnegeri* venom. The present study provided valuable phosphorylation signal transduction resources for investigating the toxic mechanism and the therapies for *Trimeresurus stejnegeri* poisoning. However, the limitations of this study are as follows: (1) there is no treatment group to study the changes of phosphorylated proteomics of the snake venom after treatment and (2) it is only a preliminary study. No more experiments have been carried out on the found differential proteins and further toxicological experiments are still needed.

## Figures and Tables

**Figure 1:** The image of PCA. The correlation between the control group and model group is described from different dimensions. Each dot represents the result of one repeat and the color represents different groups. Control: CK1, CK2, CK3. Model: M1, M2, M3.

**Figure 2:** The volcano plots of differentially expressed proteins. In the abscissa, the farther the distance to 0 point, the higher multiples of protein expressional differences were observed on the protein expression. On the ordinate, the farther the distance from 0 point, the more significant difference was observed in the protein expression. The red dots represent upregulation and blue dots represent downregulation. The gray dots represent proteins with no significant expression difference.

**Figure 3:** The bar chart of enrichment and distribution of biological processes of differentially expressed proteins in two groups. The functions of differentially expressed proteins are mainly involved in the following biological processes: immune response, regulation of blood coagulation process, intracellular ion homeostasis, regulation of complement activation, and positive regulation of cellular transcriptional translation.

**Figure 4:** The image of KEGG pathway enrichment analysis on differentially expressed proteins between the control and the model group. Entries with larger bubbles contained more differentially expressed proteins. The *p* value became smaller as the color of bubble changed from red-green-blue-purple, which indicated more significant differences.

**Figure 5:** PPI analysis on differentially expressed proteins. The circle represents the differentially expressed proteins and the size of circles represents the degree of connectivity between two proteins. PPIs involved in differentially expressed proteins mainly focused on hemolysis proteins, immune regulatory proteins, and extracellular matrix regulatory proteins.

**Figure 6:** The expression level of TF, p-TF, SLC16A1, and p-SLC16A1 was evaluated by the Western blot assay. Compared to the control group, p-TF/TF was significantly upregulated in the model group. In addition, compared to control, the expression level of p-SLC16A1/SLC16A1 was found significantly suppressed in the model group (*p* < 0.05).

**Table 1:** The concentration of isolated proteins.

Sample name	CK1	CK2	CK3	M1	M2	M3
Concentration (*μ*g/*μ*L)	18.4	16.6	17.6	16.4	13.3	13.7
Volume (*μ*L)	500	500	500	500	500	500

Control: CK1, CK2, CK3; Model: M1, M2, M3.

## Data Availability

The data used to support the findings of this study are available from the corresponding author upon request.
